This article has been retracted.

# Construction of College Students' Employment Quality Evaluation Model System under the Background of Digitalization

**DOI:** 10.1155/2022/4368369

**Published:** 2022-09-20

**Authors:** Shiming Li, Jun Jiang

**Affiliations:** College of Educational Sciences, Harbin Normal University, Heilongjiang, Harbin 150025, China

## Abstract

In the era of knowledge economy, human resources are being valued by various countries and regions. The report of the 19th National Congress of the Communist Party of China pointed out that “talent is a strategic resource for realizing national rejuvenation and winning the initiative of international competition. We must adhere to the principle of the party's management of talents, gather talents from all over the world and use them, and accelerate the construction of a strong country with talents.” College students are an important part of talents, and their employment intentions directly affect employment behavior. With the development of education in our country, the enrollment quota of most colleges and universities in the country has gradually increased, and the number of graduates has also increased. Social and economic development has different needs for different professional and technical personnel, and the employment situation in different regions is uneven. Under the increasingly complex employment environment, college students have to face greater employment pressure and compete with each other in a narrower employment field. Therefore, it is necessary to conduct better employment guidance and employment quality evaluation for college students. Based on the improved algorithm of BP network, an artificial intelligence-based employment quality evaluation model is constructed. The design model is optimized by introducing a momentum variable factor, adjusting the learning rate and quasi-Newton method, and training and recommending each optimization model through the training data. The experimental results show that the iterations of the gradient descent algorithm and the additional momentum optimization algorithm are far more than 1000 times. Second, the optimal validation errors of the two algorithms are large and the model performance is poor. The quasi-Newton ring algorithm also has faster coordination speed, stronger stability, and better overall performance. The adaptive learning rate optimization algorithm is performed in these 4 algorithms. In terms of accuracy, the accuracy of the adaptive learning rate BP optimization algorithm is 76.4%, followed by the Newton algorithm and the additional momentum algorithm, and the gradient descent algorithm is the worst.

## 1. Introduction

In recent years, with the deepening of the aging society, the reduction of labor supply, and the structural shortage in the labor market, how to retain people and how to retain more high-quality talents have become the key to improving the core competitiveness of the city.. Local governments have introduced the “New Talent Policy” one after another, providing support in terms of minimum wage commitments, rent subsidies, housing subsidies, living subsidies, etc., and provide all-round guarantees, in order to improve the city's attractiveness and attract talents. With the number of graduates waiting to be employed or unemployed is gradually increasing or is becoming the norm in society. The ensuing employment difficulties for college students have gradually become the focus of social concern and a hot issue in the field of higher education research. At present, society and high schools pay more attention to the employment rate of college students, which is a quantitative indicator. The definition of “employment rate” is clear, and the calculation is simple. It can explain the employment rate at a certain level for graduates of certain high schools and certain majors. The relationship between supply and demand in the market can also reflect the cultivation of talents in colleges and universities. However, a single “employment rate” cannot reflect the complex employment status of graduates, such as graduates' employment level, employment structure, and occupational matching, nor can it fully and objectively reflect the quality of education and teaching in colleges and universities. Therefore, it is of great significance to explore the establishment of a comprehensive, scientific, and reasonable evaluation system for the “employment quality” of college graduates.

Any scholar has put forward his own understanding and opinions on the employment quality issues in their respective fields. Wang Quanzhang started from four dimensions: employment conditions, development space, labor relations, and welfare and security were established as the first-level indicators. In these four areas, there are 15 secondary indicators, such as labor compensation, working hours, work, and environment and professional peers [1]. Liu started to establish an innovative evaluation method of 5 first-level indicators, 17 second-level indicators, and 5 third-level indicators from five aspects and adopted Delphi's method of soliciting expert opinions to screen the indicators to ensure the accuracy of employment data. The formulation and research methods of the employment quality evaluation system for college graduates studied by some scholars were evaluated [2]. Li also uses the Delphi expert method to screen the research indicators and uses the fuzzy comprehensive evaluation method and weighting algorithm to determine the final evaluation value. Under the employment policy and system, there are also four tertiary indicators [3]. There is a certain relationship between the quality of employment and “decent work.” “Provide decent, productive and sustainable employment opportunities for men and women in conditions of freedom, equity, security and human dignity. The pursuit of decent work mainly includes “protection of rights, employment, social security and fair dialogue at work.” This is an important goal [4]. Sachs uses pre-employment job and professional matching, and post-employment work attitude to evaluate employment quality [5]; Rudolph uses overall job satisfaction, professional requirements for specific jobs, and school rewards to evaluate the employment quality of graduates [6]; Arellano used innovation and entrepreneurship indicators to study the impact of graduate employment quality evaluation [7].

In recent years, with the increasing maturity and development of artificial intelligence, artificial intelligence has achieved very successful applications in the fields of big data computing, face recognition, data processing, etc., but it is rarely used in employment quality evaluation models. Through the construction of BP neural network and three improved algorithms, four artificial intelligence-based evaluation models of college students' employment quality are proposed, which can effectively improve the evaluation efficiency and accuracy of the evaluation models of college students' employment quality.

## 2. Related Work

Foreign scholars have studied the employment of college students earlier. Schomburg Harald believes that the transition from student status to work status requires a process. The vast majority of college students find their first job within six months or even longer after graduation. The work they do during school is not closely related to their majors, and low wages are becoming more and more common. Li and others believe that there are three factors that affect the employment rate of college students, namely, the scholarship rate of colleges and universities, the education expenditure of each student, and the number of students per teacher. It can be seen that college students are facing certain employment pressure. There are many studies on employment intention abroad. Holland put forward the personality type theory of personality and career matching, which is the most influential career choice theory in the field of foreign employment intention research. He believes that career choice is an extension of personal personality. He divided personality into six types: practical, research, artistic, social, commercial, and traditional. People with different personality types will be interested in the corresponding job types. This theory believes that people should take their own personality characteristics as an important standard for choosing a career. Only when the personality type is consistent with the professional characteristics, employees can obtain the best work enthusiasm. Luo's theory of psychological needs is different from this. It believes that family education has a great impact on personal career choices. Mycos college mentioned in the “College Students' employment report” that more and more college students take urban choice into consideration. In recent years, college graduates have paid more and more attention to the employment choice of cities. On the one hand, various regions have introduced talent policies to attract and retain more talents. The speed is very fast, and the gap between cities is gradually narrowing. Especially at present, many second tier cities are developing rapidly, and the gap with first tier cities is gradually narrowing. Graduates are also paying more and more attention to second tier cities, as well as broader and more employment cities.

The Hopfield network was proposed in 1980 to enable people to realize nonlinear functions by increasing the depth of the network, thus triggering the second wave of artificial intelligence research. However, the algorithm did not make a big splash at the time because its computations were easily trapped in local minima. In 1986, a breakthrough was made in neural network algorithms. A group of scientists led by Rumelhart and McCelland proposed the well-known error back-propagation (BP) algorithm [5]. The BP algorithm is a unique and attractive program, and the neural network is a challenging frontier technology, so the two are combined into a BP neural network. According to the properties and regularities of the function, the neural network can automatically learn past experience from the provided complex data samples. For complex functions, especially nonlinear functions, the advantages of neural networks can be brought into play. Neural network has the characteristics of high self-adaptation, self-organization, and self-learning. According to the laws and characteristics of functions, the neural network can scientifically and rationally analyze complex problems and find the most effective strategies and methods to solve them. For students, career guidance is a macro-information feedback process. This feedback information can not only help students make employment decisions but also provide a basis for schools to adjust their talent training models, thereby improving the overall quality of college graduates. Effectiveness of career guidance. Therefore, the employment forecast related to graduates has become a very important part of the school's employment guidance and has far-reaching significance. In foreign countries, scholars have carried out employment forecast analysis work from different aspects. Through the use of machine learning algorithms and personal historical work records, new jobs are recommended for different people; the career guidance department uses the career management service system to measure students through questionnaires and scales to objectively evaluate students' career matching. At the same time, professionals guide students online and help students develop a career direction in science.

## 3. Employment Quality Evaluation Model Based on BP Neural Network Model

### 3.1. Classical BP Neural Network

Diversity of models is a feature of artificial neural networks. According to the principle of model classification, different methods can be selected to summarize model categories. The first is the type of network topology. Different connections between neurons produce different network topologies. It is divided into a hierarchical structure, and the structure is mainly adjusted according to the level, while the interconnected structure is characterized by the close connection of each layer. The second is the type of network information flow [8]. Its structure is shown in Figure 1.

BP neural network has the following characteristics:

1. The structure of the BP neural network consists of three layers: the input layer, the hidden layer, and the output layer, and the neurons in the same layer are not connected to each other
2. The transfer function is continuously differentiable in the convergence region. In general, functions such as the unipolar sigmoid function are very classical choices
3. After the BP neural network propagates the input vector of the input layer to the hidden layer, the error finally propagated to the output layer is adjusted by the weight and continues to the input layer to continue to iterate. Through successive training iterations, the weights and thresholds are continuously adjusted until the output error is within the expected range

Standard BP neural network usually adopts gradient descent algorithm as weight training algorithm. The basic idea is that when the input signal is finally passed to the output layer, the error between the actual output and the expected output will be passed back to the input layer through the weights of the network in the next iteration. This error is actually a function, generally a mean square error function. This function takes the derivative of each dimension of the input vector and takes the derivative to zero to obtain the weight matrix. In Figure 1, the number of variables (that is, the number of feature indicators) in the input sample is *j*, the number of neurons in the hidden layer is *q*, and the number of output parameters is *m*. As shown in Figure 1, the structure diagram can determine the back-propagation neural network. The input and output expressions of the hidden and output layers of the network are the following [9–11].

1. The input to the hidden layer is:

(1) $$\begin{array}{c} {Net}_{i}=\overset{M}{\underset{j=1}{\sum }}w_{ij}x_{j}+\theta_{i}. \end{array}$$

(2) The output of the hidden layer is:

(2) $$\begin{array}{c} y_{i}=\phi \left({Net}_{i}\right). \end{array}$$

(3) The input to the output layer is:

(3) $$\begin{array}{c} {Net}_{k}=\overset{M}{\underset{j=1}{\sum }}w_{kj}x_{j}+\alpha_{k.} \end{array}$$

(4) The output of the output layer is:

(4) $$\begin{array}{c} O_{k}=\psi \left({Net}_{k}\right). \end{array}$$

The excitation function selects the unipolar function of the sigmoid function,

(5) $$\begin{array}{c} f\left(x\right)=\frac{1}{1+e^{-x}}. \end{array}$$

The defects of the standard BP neural network and its steepest descent algorithm have begun to be exposed:

1. There is no standard for the choice of network structure. So far, in the classic three-layer structure of the standard BP neural network, the number of nodes in the hidden layer has no unified standard and mathematical theory support and can only be determined based on experience and actual debugging
2. It is easy to converge to the local extreme point. The steepest descent algorithm is itself a local optimization algorithm. It is not guaranteed to find a globally optimal solution. It is easy to converge to the extreme, so that the network cannot find the optimal weights in the solution space, and ultimately, there is no better solution.
3. The convergence rate of the standard BP neural network is slow. The BP neural network adopts the fastest descending algorithm. By adjusting the weight and threshold of the network, the mean square error is propagated from the output layer to the input layer. After continuous iteration, the mean square error is reduced to the expected error range. The learning rate of the algorithm is fixed throughout the training process, and in order to ensure that the algorithm can eventually converge, the selected learning rate must not exceed the selected value. This value is also determined by experience. Therefore, the convergence rate of the standard BP neural network cannot be very fast

### 3.2. BP Neural Network and Improved Algorithm

Aiming at the problem that the fastest descent algorithm in BP neural network cannot guarantee to find the global optimal solution, it is easy to converge to the extreme point, and the optimal weight of the solution space cannot be found [12]. In this paper, momentum neural network algorithm, variable learning rate algorithm, and quasi-Newton method are selected to improve the standard of BP neural network. The specific method is as follows.

#### 3.2.1. Momentum BP Neural Network Algorithm

Momentum BP method is to add appropriate dynamic variable factors (09). When the BP neural network is trained for gradient descent, the BP neural network structure has a certain inertia: *α* < *α*<

(6) $$\begin{array}{c} \Delta w\left(n\right)=-\eta \left(1-\alpha \right)\nabla e\left(n\right)+\alpha ∆W\left(n-1\right). \end{array}$$

This formula adds the product term *α*∆*W*(*n* − 1) of the dynamic variable factor and the weight increment. This term is also known as the momentum term. It reflects the experience learned by the neural network in past iterations of training. The adjustment of the weight can play a buffering role to avoid the adjustment of the weight too fast. At the same time, the increased momentum factor is equivalent to smoothing and filtering the sequence of weight increments at each iteration, eliminating abnormal increments, and avoiding noise interference during training.

#### 3.2.2. BP Neural Network Algorithm with Variable Learning Rate

The *η* learning rate is used to adjust the convergence of the training algorithm when the neural network trains the weights and thresholds in terms of network speed. In the fastest descending BP algorithm adopted by the BP neural network, the learning rate is set as a constant. The lower the learning rate value is set, the more iterations of the training algorithm are required, and the slower the convergence to the global optimal solution; the higher the learning rate value, the faster the training algorithm oscillates on the error surface. Go back and forth to find the extremum, and it is easy to cross the extremum point. The variable learning rate BP algorithm dynamically adjusts the learning rate according to the flatness of the error surface and the ratio of the error function in a particular operation. If the error surface tends to be flat, the value of the error function gradually decreases, indicating that the output value is getting closer and closer to the expected value, indicating that the learning rate is positive at this time, and the learning rate can continue to increase; when the error surface tends to be steep, the value of the error function gradually increases. If it increases, it means that the learning rate is a negative number. It is necessary to reduce the learning rate, reduce the weight increment, and roll back the adjustment of the weight. Increasing and decreasing the learning rate can be achieved by multiplying by the factor *k*. The sign of this factor *k* can be positive or negative. If it is a positive number, it will increase the learning rate, and if it is a negative number, it will decrease the learning rate [13, 14]. The specific rules are as follows:

if (*n* + 1) < *e*(*n*),

(7) $$\begin{array}{c} \eta \left(n+1\right)=k_{inc}\eta \left(n\right), \end{array}$$

if *e*(*n* + 1) ≥ *e*(*n*),

(8) $$\begin{array}{c} \eta \left(n+1\right)=k_{dec}\eta \left(n\right). \end{array}$$

#### 3.2.3. Quasi-Newton Method BP Neural Network

The basic idea of the quasi-Newton method is to approximate the optimum point using finite or infinite differential iterations. Its basic iterative formula is as follows:

(9) $$\begin{array}{c} w\left(n+1\right)=w\left(n\right)-H^{-1}\left(n\right)g\left(n\right). \end{array}$$

*H* is the Hessian expression for the error function, which is essentially a matrix of derivative information of the error function. The quasi-Newton method only needs to calculate the differential of the objective function and does not need the information of the second derivative function. This equation approximates the second derivative, avoiding the restriction on the second derivative of the objective function. The quasi-Newton method only needs the gradient information of the objective function of the current iteration. After each iteration, the amount of calculation will be greater than the previous iteration. Even less, the convergence is much faster than the steepest descent BP algorithm.

### 3.3. Construction of Employment Quality Evaluation Model Based on BP Neural Network

#### 3.3.1. Structural Design of BP Neural Network

1. There are many nodes. The advantage is that the network has better generalization ability. The disadvantage is that it leads to slower training convergence [15–17]. In practical applications, the following estimates are usually given:

(10) $$\begin{array}{c} \overset{n}{\underset{i=0}{\sum }}C_{M}^{i}>k. \end{array}$$

(11) $$\begin{array}{c} M=\sqrt{n+m}+a. \end{array}$$

(12) $$\begin{array}{c} M=\log_{2}n. \end{array}$$

where *k* is the total number of samples, *M* is the number of neurons in the hidden layer, *n* is the number of neurons in the input layer, *m* is the number of neurons in the output layer, *a* ∈ [0, 10], if *i* > *M*, *C*_*M*_^*i*^ = 0.

(2) Design of input layer and output layer. The number of nodes in the input layer depends on the dimension of the input vector. According to the personal credit rating established in Section 2.3 of Chapter 2, for the price index system, the number of indicators designed in this topic is 17, the dimension of the input vector is 17, and the number of nodes in the input layer is 17. Since there are two classes, the output uses 1 neuron
(3) Design of transfer function. According to the research experience of the reference, in the model designed in this paper, the transfer function selects the sigmoid function unipolar function [18], namely,

(13) $$\begin{array}{c} f\left(x\right)=\frac{1}{1+e^{-x.}} \end{array}$$

#### 3.3.2. Construction of Employment Quality Evaluation Model Based on BP Neural Network

Above, we have established a system of employment evaluation indicators in colleges and universities and used the relevant indicators as the input features of the neural network model. Then, the neural network model constructed in Section 3.2 can be used to achieve end-to-end employment quality assessment in universities. According to the mathematical model of Section 3.1 of the BP network, the hidden layer formula of the employment quality evaluation model is:

(14) $$\begin{array}{c} y_{i}=f\left(\overset{17}{\underset{i=1}{\sum }}V_{ij}x_{j}\right),j=1,2,3,4, \end{array}$$

where *V*_*ij*_*v* is the weight from the input layer of the *i*th neuron to the input layer of the *j*th neuron. Therefore, after combining the sigmoid unipolar transfer function, the output layer expression of the neural network-based credit evaluation model is:

(15) $$\begin{array}{c} z=f\left(\overset{4}{\underset{j}{\sum }}w_{j}y_{j}\right), \end{array}$$

where is the weight from the input layer to the intermediate layer. In this way, formulas (13), (14), and (15) constitute a personal credit evaluation model based on the back-propagation neural network *w*_*j*_.

## 4. Experiment and Result Analysis

In this section, we will conduct simulation experiments. We compare the performance of the gradient descent algorithm with other momentum optimization algorithms, adaptive learning rate optimization algorithms, and quasi-Newton cycle algorithms in Matlab and conduct simulation experiments. At the same time, we will use the employment quality evaluation index system studied in Chapter 2, combined with the BP neural network structure designed in Section 3, to realize the employment quality evaluation model based on BP neural network in Matlab.

### 4.1. Experiment Preparation

In the German credit database, there are a total of 1000 samples, including 700 samples of applicants with good credit (positive samples) and 300 samples of applicants with poor credit (negative samples). In this simulation experiment, the first 600 positive samples and the first 200 negative samples are taken to form the training samples for this experiment, and the remaining 100 positive samples and the remaining 100 negative samples share the compose test samples for the experiment.

### 4.2. Experimental Environment

The specific experimental environments are the following:

1. The computer operating system is Windows 10
2. The configuration of the computer processor is Intel(R) Core(TM) i5-3230M CPU, 2.60 GHz
3. Memory configuration: 4 GB
4. Matlab version: R2020a (8.3.0.532), 64-bit

### 4.3. Experimental Steps

1. Prepare the experimental data and store it in an Excel file, write code in Matlab software to read the data in the file Thesis_GermanCreditData.xlsx
2. Divide the sample data set into positive samples with good credit and negative samples with poor credit
3. Prepare the training sample set and the test sample set to prepare for training the neural network
4. Create a back-propagation neural network and design four different training functions to compare and test the performance of the model designed in this experiment. The four training functions are gradient descent algorithm, additional momentum optimization algorithm, adaptive learning rate optimization algorithm, and quasi-Newton ring algorithm. In this experiment, combinations of different hidden layers are tested during the experiment. The number of hidden layer nodes can be flexibly modified according to the actual situation
5. Test the neural network to check the prediction accuracy of the model

### 4.4. Experimental Results

The experiment was divided into four groups. Under the condition that other parameters and dataset settings remain unchanged, replace the training algorithm to train the network and use the same test dataset to test the trained network model to check the performance of the model and achieve the best performance error, maximum calibration The larger the error, the worse the performance; the smaller the optimal calibration error, the better the performance of the model (the green dotted line); the target represents the target error level, i.e. the grey dotted line. Here are the model performance curves for these four experiments:

As can be seen from Figure 2, when the gradient descent algorithm is used as the training algorithm, the best verification error difference achieved is 0.147, a total of 16983 iterations are required, and the curve is relatively smooth. It can be seen that the performance curve is indeed orientable at any point.

It can be seen from Figure 3 that when the additional momentum optimization algorithm is used as the training algorithm of the BP neural network, the minimum validation error of 0.136 can be achieved, and the number of iterations is 8103. Compared with the gradient descent algorithm, it is indeed a big improvement, because it is an improved algorithm based on the gradient descent algorithm, and the performance curve is still very smooth and controllable at any time.

As can be seen from Figure 4, the adaptive learning rate optimization algorithm is used as the training algorithm of the BP neural network. This method can achieve a minimum verification error of 0.12, which are both the performance of the gradient descent algorithm and the performance of the additive momentum optimization algorithm. To be better, it only takes 135 iterations and is faster.

It can be seen from Figure 5 that the iteration efficiency of the quasi-Newton ring algorithm is very high, and only 4 iterations are required. The best calibration error is 0.178, and the model performance is not bad.

Based on the model performance of the above four BP neural network training algorithms, the summary experimental results are shown in Table 1:

In Table 1, the best validation error represents the validation of the trained model using the test dataset. The smaller the value, the better the performance of the algorithm model. It can be seen from Table 1 that the number of iterations of the gradient descent algorithm and the additional momentum optimization algorithm is much greater than 1000, the optimal verification error of the two algorithms is large, and the model performance is poor. The quasi-Newton ring algorithm also has a faster convergence rate, stronger stability, and better overall performance. The adaptive learning rate optimization algorithm is performed in the middle of these four algorithms.

In terms of accuracy, when these four training algorithms are applied to personal credit evaluation, the additional momentum BP optimization algorithm has the lowest prediction accuracy of 70.4%, and the adaptive learning rate BP optimization algorithm has an accuracy of 76.4%, indicating the learning rate. The influence in the gradient descent algorithm is very large. The accuracy of the quasi-Newton algorithm is 72.8%. Overall, the prediction accuracy of the college student employment quality evaluation model based on BP neural network exceeds 70%.

## 5. Conclusion

As an advantageous group in the labor market, college graduates are the main force to enhance the city's innovation ability, promote industrial upgrading, and enhance the city's core competitiveness. The flow and distribution of their employment is of great significance to the development of the region. Although many cities have introduced preferential policies to retain graduates, many college students still show a trend of outflow in their choice of employment location. So what are the factors that college students consider when choosing a place of employment and what are the factors that affect the employment of college students in their place of study? According to the commonalities and characteristics of the employment status of various colleges and universities, this research constructs the overall evaluation index of the employment quality of various colleges and universities and builds the employment quality evaluation model based on the neural network based on the improved algorithm of the BP network. The main work is as follows:

1. According to the comprehensiveness, simplicity and operability of the employment quality evaluation system in colleges and universities, combined with the commonality and characteristics of various colleges and universities, construct efficient and general evaluation indicators, which are mainly used in the evaluation index system of employment quality in colleges and universities.
2. On the basis of analyzing the BP neural network algorithm under the artificial intelligence network algorithm, the structure design of the BP neural network based on the gradient descent algorithm is constructed, and the design model is optimized by introducing the momentum variable factor, and the learning rate and simulation are carried out. The results show that the neural network model proposed in this paper can evaluate the employment quality of colleges and universities more comprehensively

## Figures and Tables

**Figure 1:** Basic structure model of BP neural network.

**Figure 2:** Gradient descent algorithm—Train-d.

**Figure 3:** Additional momentum optimization algorithm—Train-dm.

**Figure 4:** Adaptive learning rate optimization algorithm—Trinda.

**Figure 5:** Quasi-Newton ring algorithm—Train-bfg.

**Table 1:** Performance comparison of training functions.

Training algorithm	Train-gd	Train-gdm	Train-gda	Train-bfg
Number of iterations	16983	8097	135	4
Best calibration error	0.147	0.136	0.122	0.178
Accuracy	0.716	0.704	0.764	0.728

## Data Availability

The dataset can be accessed upon request.
